The article "Experimental Study of Local Inner Ear Gene Therapy for Controlling Autoimmune Sensorineural Hearing Loss" was retracted in 2017. Reasons: duplicated images; concerns about the data.

# Experimental Study of Local Inner Ear Gene Therapy for Controlling Autoimmune Sensorineural Hearing Loss

**DOI:** 10.1155/2014/134658

**Published:** 2014-04-07

**Authors:** Chang-qiang Tan, Xia Gao, Wen-jun Cai, Xiao-yun Qian, Ling Lu, He Huang

**Affiliations:** ^1^State Key Laboratory of Materials-Oriented Chemical Engineering, College of Biotechnology and Pharmaceutical Engineering, Nanjing University of Technology, No. 5 Xinmofan Road, Nanjing, Jiangsu 210009, China; ^2^Nanjing Drum Tower Hospital, The Affiliated Hospital of Nanjing University Medical School, Jiangsu 210008, China; ^3^Department of Otolaryngology, Affiliated Zhongda Hospital of Southeast University, Nanjing, Jiangsu 210009, China

## Abstract

This study aimed to investigate the efficacy of gene therapy for treating autoimmune sensorineural hearing loss (ASHL) via local administration of a recombinant adenovirus vector containing the Fas ligand or interleukin IL-10 gene. Guinea pigs were divided into four groups, with different microinjections in the scala tympani. Group A were injected with FasL-EGFP, B with IL-10-EGFP, C with EGFP, and D with artificial perilymph. Seven days later, auditory brain-stem response (ABR) was tested, and the temporal bone was stained and observed by light microscopy. The spiral ligament and basement membrane were observed using transmission electron microscopy. FasL and IL-10 expression were examined using immunofluorescence histochemistry. Immunohistochemical analysis showed that the recombinant adenovirus vector in Groups A, B, and C can transfect the stria vascularis, the spiral ligament, the organ of Corti, the spiral ganglion, the region surrounding the small blood vessel in the modiolus, and the cochlear bone wall. Compared with those in Groups C and D, the ABR wave III mean thresholds were significantly lower and the inner ear immunoinflammatory responses in Groups A and B were significantly alleviated. Inhibition of immunoinflammatory response alleviated immunoinflammatory injury and auditory dysfunction. This technique shows potential as a novel therapy for ASHL.

## 1. Introduction

Based on the clinical finding that 18 patients with hearing disorders significantly improved after immunosuppressive therapy, McCabe [1] proposed the concept of autoimmune sensorineural hearing loss (ASHL) in 1979. Further research showed that autoimmune damage not only affected the cochlea, but also spread to the vestibule; autoimmune inner ear disease was subsequently described [2]. Although many studies have advanced our understanding of hearing loss caused by this disease, the etiology and pathogenesis of ASHL remain unclear. Specific clinical diagnostic methods are lacking, and problems have arisen with therapies for ASHL patients, owing to the toxicity and side effects of corticosteroids and immunosuppressive therapy and a relatively high relapse rate despite an improved efficacy and more rapid response to treatment.

With the development of molecular biology and genetic engineering technologies, gene therapy has become a hot topic for therapeutic research. Lalwani et al. [3] and Raphael et al. [4] reported gene introduction into the inner ears of animals in 1996. Since then, gene therapy in the inner ear has become the focus of much research, and great progress has been made in the choice of vectors, methods of introduction, and procedural safety [5]. Genetic engineering allows the construction of a vector that can carry therapeutic genes into the animal inner ear, without virus-associated ototoxic reactions, making gene therapy for ASHL possible. In addition, Fas ligand (FasL) and interleukin-10 (IL-10) are commonly involved in autoimmune diseases and are therapeutically effective as the targets of gene therapy [6–14].

Replication-defective adenoviral vector is safe and effective, with a high virus titer, high transfection efficiency (100%), and enormous capacity for carrying exogenous genes. It does not integrate with host chromosomal DNA, which eliminates the possibility of hazardous insertion mutations. It is also stable and can be easily prepared and purified. In addition, adenoviruses characteristically infect a wide range of host cells, including both mitotic-phase cells and nonmitotic-phase terminally differentiated cells. Adenoviral vector is therefore one of the most frequently applied vectors in gene transduction studies. Yagi et al. [15] and Husseman and Raphael [16] introduced gene-carrying viruses into the scala tympani through the round window membrane and reported that the gene product was subsequently expressed and functional in the cochlea.

Based on these reports, we conducted an experimental study on gene therapy for autoimmune suppression or regulation in the inner ear of ASHL-model animals and explored the therapeutic efficacy and possible side effects of local inner ear treatment.

## 2. Materials and Methods

### 2.1. Experimental Animals

Healthy mature albino guinea pigs with white hair and red eyes (Dunkin Hartley), weighing approximately 300 g, were selected. They had normal auricular reflexes and underwent otoscopy to exclude middle ear disorders at the Experimental Animal Center of Nanjing Medical University (China). This study was carried out in strict accordance with the recommendations of the Regulations on the Management of Laboratory Animals of the State Scientific and Technological Commission of China. The protocol was approved by the Committee on the Ethics of Animal Experiments at Nanjing Medical University (Permit number SCXK (Sue) 2007-0008). All surgical procedures were performed under sodium pentobarbital or ether anesthesia, and all procedures involving animals and their care conformed with institutional guidelines, which were in compliance with national and international laws and guidelines.

### 2.2. Preparation of Guinea Pig Inner Ear Antigens (IEAgs)

Guinea pigs IEAgs were prepared as described previously [17]. Briefly, a guinea pig was decapitated under ether anesthesia and the temporal bone was removed; the bulla was opened immediately, and the membranous labyrinth, including the basement membrane, spiral ligament, membranous semicircular canals, utricle, and saccule (to remove the otolith apparatus), was isolated under a dissecting microscope; it was then placed in phosphate-buffered saline (PBS) solution of 0.01 mol/L with pH 7.4. After tissue grinding, ultrasonic crushing, homogenisation, and centrifugation (1000 r/min, 5 min), the supernatant was used to assay protein content with an ultraviolet spectrophotometer. The IEAgs solution was dispensed into vials (2 g protein per vial) and freeze-dried; the dry IEAgs powder for experimentation was refrigerated at −80°C.

### 2.3. Preparation of ASHL-Model Animals

IEAgs at 400 mg/0.4 mL were used for the first immunization of the animals and were injected into the right rear footpad with an equal amount of complete Freund's adjuvant (Ad). A multipoint subcutaneous dorsal injection of IEAgs (200 mg/0.4 mL) and incomplete Ad was administered 2 weeks later. An identical immunization was administered 2 weeks later. ASHL-model animals were identified based on the elevation of wave III threshold (greater than the mean value plus 2 standard deviations of preimmunization measurements in all animals) in their auditory brainstem response (ABR) and the appearance of IEAg-specific antibodies (*A* value at a wavelength of 490 nm was greater than the mean value plus 2 standard deviations of preimmunization measurements in all animals, determined with an ELISA) [17].

### 2.4. Recombinant Adenovirus Construction

#### 2.4.1. Construction of Recombinant Gene Vector

The recombinant gene vector was constructed by the Shanghai DoBio Biotech Co., Ltd. (China), using the plasmids pAV.Ex1d-CMV>IL-10/IRES/EGFP and pAV.Ex1d-CMV>FasL/IRES/EGFP and the genes IL-10 and FasL. IL-10 and FasL were cloned into the adenovirus vector plasmid PAdTrack-CMV using PCR cloning technology. Homologous recombination was performed with plasmid backbone sequences in* E. coli Stbl3* cells. Recombinant adenoviral vectors, Ad-IL-10-EGFP and Ad-FasL-EGFP, were obtained after packaging and amplification in HEK293 cells, and the EGFP marker gene was packaged.

#### 2.4.2. Identification and Purification of the Recombinant Gene Vectors

*(1) RT-PCR.* Recombinant plasmid-transfected HEK293 cells and their supernatants were collected, and viral DNA was extracted as a template. PCR amplification was performed with IL-10 and FasL primers. The primers for PCR amplification of the IL-10 and FasL target genes were designed according to a cDNA expression library, and their exact sequences are as follows: IL-10-Agel-F: 5′-GAGGATCCCCGGGTACCGGTCGCCACCATGCCTGGCTCAGCACTG-3′, IL-10-Agel-R: 5′-TCACCATGGTGGCGACCGGGCTTTTCATTTTGATCATCATG-3′, FasL-F: 5′-CTGGGGATGTTTCAGCTCTTC-3′, and FasL-R: 5′-CTTCACTCCAGAAAGCAGGAC-3′. The recombinant plasmids were identified using colony PCR and sequencing with the following primers: EGFP-N-5: 5′-TGGGAGGTCTATATAAGCAGAG-3′; EGFP-N-3: 5′-CGTCGCCGTCCAGCTCGACCAG-3′. Electrophoresis of the plasmids showed bands of specificity at 540 bp and 296 bp, as expected for the IL-10 and FasL genes (Figure 1).

After DNA sequencing, the confirmed plasmids were extracted using a plasmid DNA mini-preparation kit according to the manufacturer's instructions (Qiagen, US) and were identified using 1% agarose gel electrophoresis. The plasmid concentration was evaluated using an ultraviolet spectrophotometer.

*(2) Virus Purification and Virus Titer Determination.* Virus purification was conducted using an adenovirus purification kit (Biomiga, USA), according to the manufacturer's instructions. Virus titers were determined using plaque assays. In brief, HEK293 cells were seeded onto 24-well plates. When grown to 90% confluence, HEK293 cells were infected with a series of virus dilutions (ranging from 10^1^ to 10^12^) until plaque formation began. The virus titer (plaque forming unit (PFU)/mL) was calculated using the following formula: virus titer = (number of plaques × dilution)/volume of diluted virus added to the well. 

*(3) Observation of Transfected 293T Cells with Fluorescence Microscopy. *HEK293T cells were transfected with Ad-IL-10-EGFP or Ad-FasL-EGFP recombinant adenovirus vector. Both types of cells showed strong fluorescence reactions (Figure 2).

### 2.5. Experimental Design

Thirty-two ASHL-model animals were randomly divided into four groups of eight animals each; the animals received injections in the scala tympani as follows: Group A received Ad-FasL-EGFP, Group B received Ad-IL-10-EGFP, Group C received Ad-EGFP, and Group D (control group) received artificial perilymph (NaCl 125 mM/L, KCl 3.5 mM/L, NaHCO_3_ 25 mM/L, NGGL_2_ 1.20 mM/L, NaH_2_PO_4_ 0.75 mM/L, CaCl_2_ 1.3 mM/L, and glucose 5.0 mM/L, with pH 7.4).

### 2.6. Technique for Microinjection of Recombinant Gene Vector into the Tympani

Microinjection was performed 2 weeks after the final immunization. Guinea pigs were anesthetized by intraperitoneal injection of 1% sodium pentobarbital (30 mg/kg). An incision of approximately 3-4 cm was made behind the auricle to expose the bulla; a miniature electric drill was used to open the bulla to expose the cochlear turn; the cochlear bony wall of the scala tympani near the round window niche was gently ground until thin, and then a pinpoint size of the hole was drilled. The tip of a pediatric scalp intravenous needle was inserted into the scala tympani (i.e., perilymph lacuna) to a depth of no more than 1 mm with a microthruster, and a small amount (approximately 10 *μ*L) of perilymph was drawn out. The recombinant adenovirus vectors or artificial perilymph was injected into the scala tympani with a microinjector; Group A received 20 *μ*L Ad-FasL-EGFP (virus titer of 2.5 × 10^10^ pfu/mL), Group B received 20 *μ*L Ad-IL-10-EGFP (virus titer of 1.0 × 10^8^ pfu/mL), Group C received Ad-EGFP (virus titer of 1.0 × 10^9^ pfu/mL), and Group D received 20 *μ*L artificial perilymph. The hole in the bone at the turn of the cochlea was sealed with bone wax and the skin incision was sutured. All operations were strictly in compliance with aseptic principles.

### 2.7. Observational Index

#### 2.7.1. Specific Immune Reaction Assay

Specific antibodies against IEAgs were assayed by ELISA, which was performed before immunization and 2 weeks after the last immunization. Blood from the heart was collected and the serum was separated and collected. Each well of the ELISA plate was coated with 100 *μ*g/mL IEAgs solution, sealed, and stored overnight at 4°C. Guinea pig serum was diluted 1 : 10 and aliquoted into each hole using a Finnpipette (Thermo Scientific, China) and incubated at 37°C for 2 hours. The plate was washed 4 times and horseradish peroxidase-labeled Staphylococcal protein A-HRP (SPA-HRP) diluted 1 : 2000 was aliquoted into each hole with a Finnpipette and incubated at 37°C for 1 hour. The plate was washed 4 times and H_2_SO_4_ was added after 10 minutes to halt the coloration, using* ortho*-phenylenediamine-hydrogen peroxide solution as the substrate. The absorbance value (*A*) at a wavelength of 490 nm was measured using an ELISA reader.

#### 2.7.2. ABR Test

An ABR test was performed one week before immunization, two weeks after the last immunization, and one week after the tympanic injection. A pin-shaped test electrode was inserted at the junction of the coronal and sagittal sutures in each guinea pig's head, while a reference electrode was subcutaneously inserted near the mastoid tip, behind the pinna, and a grounding electrode was subcutaneously inserted into the nasion. The repetition frequency of the click stimulus signal was 11 times/min, superimposed 2048 times with a 10 ms recording duration. The threshold of wave III was measured.

#### 2.7.3. Microscopic Observations of the Inner Ear

Two guinea pigs in each group were decapitated under anesthesia for immediate removal of the temporal bone after the hearing test; their bulla was opened and placed in 4% paraformaldehyde fixative for 24 hours, placed in 10% ethylene diamine tetraacetic acid (EDTA) for 7–10 days for decalcification, and then soaked in lithium sulfate for 24 h (to prevent tissue swelling). After gradual alcohol dehydration, gum dipping, directional collodion embedding, and block repairing, 25 *μ*m slices were cut with a level slicer. Three slices taken from near each modiolus were preserved in 70% alcohol for HE staining and observation under a light microscope.

#### 2.7.4. Immunohistochemical Analysis

*(1) Inner Ear Paraffin Slices.* Four guinea pigs in each group were decapitated under anesthesia for immediate removal of the temporal bone after the hearing test; their auditory vesicles were opened and placed in 4% paraformaldehyde fixative. The round window niche was opened and several injections were performed through a small hole drilled in the cochlear tip and fixed for 24 hours; they were decalcified for 7–10 days in 10% EDTA and washed for 1-2 hours after fixing. Standard dehydration, transparency, wax dipping, directional embedding, and continuous slicing (5 *μ*m thickness) were performed, as previously described.

*(2) Immunofluorescence Analysis.* Three modiolus slices were selected for bleaching, fishing, and sticking, and after conventional dewaxing they were placed under an inverted fluorescence microscope (fluorography) for observation and photography. 

*(3) Immunohistochemical Analysis.* Antigen repair was performed to obtain slices with 0.2% trypsin. After blocking for 10 min with goat serum, the first antibody, diluted in PBS, was added (Group A received rabbit anti-mouse (RAM) FasL, Group B received RAM IL-10, and Groups C and D received RAM FasL and IL-10); preparations were incubated overnight at 4°C. The second antibody, SPA-HRP, was added and incubated for 30 min at 37°C after washing 3 times with PBS for 5 min. Following additional three rounds of washing with PBS for 5 min, DAB staining, slide sealing, and optical microscopic observations were performed, and photographs were taken. 

*(4) Transmission Electron Microscopy (TEM).* Two guinea pigs in each group were decapitated under anesthesia for immediate removal of the temporal bone following the hearing test; after fixation in 2.5% glutaraldehyde, the total internal membranous labyrinths (spiral ligament, basilar membrane) were removed and washed in 0.1 M phosphate buffer (PB). Samples were postfixed in 1% osmium tetroxide for 2-3 hours, dehydrated in ethanol, and embedded in 100% acetone. Ultrathin sections were sliced using a Reichert Ultracut E ultramicrotome, stained with uranyl acetate and lead citrate, and examined using a Philips CM10 transmission electron microscope at 80 kV.

## 3. Results

### 3.1. Specific Immune Response Test Results

Antibody levels were significantly elevated after immunization and inner ear injection in all experimental groups and in the control group treated with IEAgs, and significant differences were observed among the preimmunization, postimmunization, and post-inner-ear-injection groups (*t*-test, *P* < 0.05, Table 1). No significant differences were observed within the preimmunization, postimmunization, or post-inner-ear-injection groups (*t*-test, *P* > 0.05).

### 3.2. Auditory Function

The ABR wave III reaction threshold was used as an indicator of hearing level, and the results are shown in Table 2 and Figure 3. The postimmunization mean ABR threshold was higher in each group than the preimmunization threshold, and significant differences were observed within each group (*t*-test, *P* < 0.05). Means of the ABR thresholds after inner ear injection in experimental Groups A and B were lower than after immunization, and significant differences were found within each group (*t*-test, *P* < 0.05). The ABR threshold mean in Group A was lower than that of Group B (*t*-test, *P* > 0.05). There was no significant difference between Group C and Group D before and after inner ear injection. There was no significant difference between the right and left ears within each group (*t*-test, *P* > 0.05).

The postimmunization ABR threshold mean of wave III minus 2 standard deviations was used as the criterion for judging auditory function improvement in Groups A and B. Auditory function in Group A (7 ears of 4 guinea pigs) and Group B (5 ears of 3 guinea pigs) was greatly improved after inner ear injection, with a therapeutic efficacy of 38.89% (7/18) and 27.78% (5/18) in Groups A and B, respectively. Similarly, the postimmunization ABR threshold mean of wave III minus 2 standard deviations was used as the criterion for judging auditory function improvement in Groups C and D. No significant difference in auditory function was found between the groups after local inner ear injection (*t*-test, *P* > 0.05).

### 3.3. Microscopic Observation of the Inner Ear

A significant inner ear inflammatory reaction occurred in Groups C and D (Figures 4, 5, and 6), including the infiltration of Rosenthal's tube with inflammatory cells (primarily mononuclear cells). Spiral ganglion cell degeneration (primarily cell body swelling) and decreased spiral ganglion cells were observed in some animals compared with the control group. In some animals, hemosiderin deposition in the stria vascularis, floccules in the cochlear duct, scala tympani, or vestibuli and “floating cells” in the cochlear duct were observed, but no significant abnormalities were observed in the organ of Corti. In Groups A and B, the inflammatory reaction was significantly less severe than in Groups C and D, especially in the improvement of auditory function. Some mononuclear cell infiltration was observed in the perivascular modiolus only, but no abnormalities of spiral ganglion cells were observed; no obvious abnormalities were observed in the organ of Corti or the stria vascularis. Some floccules were found in the scala tympani, but “floating cells” were absent.

### 3.4. Immunohistochemical Analysis

#### 3.4.1. Immunofluorescence Histochemistry

Fluorescence display did not differ markedly between Groups A, B, and C; fluorescence was primarily distributed in the cochlear bone wall, the inner lip of the cochlear duct in the spiral plate, the spiral ligament, the stria vascularis, and so forth. No significant accumulation of fluorescence was observed in the inner ear tissues of Group D (Figures 7, 8, and 9).

#### 3.4.2. Immunohistochemical Analysis

Immunohistochemical analysis showed that the primary color reactions (FasL expression) could be observed in the spiral ganglion, organ of Corti, vascular pattern, perivascular modiolus, cochlear bony wall, ampullary crest, and other organs in Group A animals (Figures 11, 13, and 14). The main sites of color reaction (i.e., IL-10 expression) in Group B (Figure 12) included the stria vascularis, spiral ligament, organ of Corti, spiral ganglion, and cochlear bony wall, whereas only weak coloration was observed in the spiral ganglion and cochlear bony wall in Groups C (Figure 10) and D.

### 3.5. TEM Observations

No particular pathologic changes were observed in the cells or intracellular structures of animals in any group; mitochondrial swelling was observed within the epithelial cells of the stria vascularis in Group C only (Figures 15 and 16).

## 4. Conclusion

Although the pathogenesis of ASHL remains unclear, research on autoimmune diseases and their pathological changes indicates that several cytokines play important roles. Studies have reported that anti-inflammatory molecules such as IL-10 [18, 19] show efficacy in animal-model gene therapy—for example, in the prevention of autoimmune disease, such as rheumatoid arthritis, multiple sclerosis, and autoimmune thyroiditis. Whether the pathogenesis of ASHL is characterized by cellular or humoral immunity remains unclear. Given its proapoptotic activities on T lymphocytes [20], the FasL gene was selected as a therapeutic target for ASHL to explore the regulatory effects of gene therapy on cellular immunity. The introduction of a constructed adenovirus into the cochlea reportedly results in the successful expression of its contained gene in the guinea pig cochlea without physiological inner ear dysfunction [4, 21].

We have successfully developed an ASHL-animal model [16]. After IEAgs immunization of guinea pigs, the present study successfully produced ASHL animals with elevated levels of specific antibodies in their serum; that is, an ASHL animal model was obtained. Ad-FasL-EGFP and Ad-IL-10-EGFP were introduced into the inner ear of guinea pigs via scala tympani fenestration and microinjection technology. ABR testing was performed to examine the auditory functions of the experimental animals, fluorescence microscopy was used to assess virus transfection into the inner ear, and enzyme immunohistochemistry was performed to observe the expression of gene products.

The results showed that auditory function was significantly improved in some experimental animals (i.e., their ABR wave III threshold was lowered) after local injection of a recombinant adenovirus vector carrying an immunomodulatory gene. A significant difference was observed between experimental groups and the control group in terms of mean threshold within groups. Inner ear pathological tissue morphology indicated that immune inflammatory reactions were weaker in two of the experimental animal groups than in the control group. Floccules were observed in the cochlear duct of only a few experimental animals, and no changes were observed in spiral ganglion cells. The stria vascularis and organ of Corti were essentially normal, indicating that local immunomodulatory gene therapy was efficacious; it controlled inflammation and injury in the inner ear, reversing lesions and improving auditory function. To date, the characteristics and nature of the floating cells that appear in the cochlear duct remain unknown and require further study. Enzyme immunohistochemistry results show that recombinant adenovirus introduced into the inner ear (perilymphatic space) was successfully transfected and was primarily distributed in the cochlea bony wall, the cochlear duct within the bone spiral lamina lip, and the spiral ligament and stria vascularis. FasL gene expression products were primarily distributed in the spiral ganglion, organ of Corti, stria vascularis, perivascular modiolus, cochlear bony wall, and ampullary crest. IL-10 gene expression products were primarily distributed in the stria vascularis, spiral ligament, organ of Corti, and cochlear bony wall. Taken together, these results suggest that a single scala tympani injection becomes widely distributed through various tissues in the inner ear. Given the inner ear's anatomy and histology, we speculate that distribution of the adenovirus from the scala tympani to the cochlear duct can be attributed to three pathways: (1) connection with the tympanic perilymph through small holes under the bone spiral lamina; (2) connection with tympanic perilymph through small holes in cochlear nerve fibers; (3) the fact that the scala tympani can be connected with the scala vestibuli through the helicotrema at the cupulae cochleae and endolymph in the cochlear duct interchanging with the perilymph through the vestibular membrane.

Intriguingly, immunohistochemical analysis of Groups A and B showed significant viral transfection and expression of immunomodulatory gene products in the cochlea bony wall; however, the mechanism remains unclear. As reported in previous studies, obvious inflammatory lesions (which were very similar to sclerosis bone lesions, thus supporting the autoimmune etiological hypothesis for this disease) were found in the cochlea bony wall after IEAgs immunization in guinea pigs. Whether this type of gene therapy also affects autoimmune otosclerosis will be confirmed through further studies.

The injection of Ad-EGFP into ASHL animals in one experimental group produced no significant changes in auditory function, and the pathomorphological changes observed in the inner ear were similar to those in the control group, in which artificial perilymph was injected. This result indicates that the adenovirus caused no additional damage or physiological dysfunction to the inner ear and produced no obvious therapeutic effects in ASHL.

## Figures and Tables

**Figure 1:** Reverse transcription polymerase chain reaction analysis of human embryonic kidney (HEK) 293T cells with interleukin-10 (IL-10; 540 bp) (a) and Fas ligand (FasL; 296 bp) (b) messenger RNA expression.

**Figure 2:** HET293T cells transfected with Ad-IL-10-EGFP (a) and with Ad-FasL-EGFP (b) showed a fluorescence reaction (20 × 10). Ad: Freund's adjuvant; EGFP: enhanced green fluorescent protein.

**Figure 3:** (a) Auditory brainstem response (ABR) waveform of an animal in Group A before immunization. Arrows indicate that the hearing threshold of wave III is less than 30 dB (sound pressure level (SPL)). (b) ABR waveform of the same animal after immunization. Arrows indicate that the hearing threshold of wave III is 70 dB (SPL). (c) ABR waveform of the same animal 2 weeks after gene therapy. Arrows indicate that the hearing threshold of wave III is less than 50 dB (SPL).

**Figure 4:** photograph of a spiral ganglion slice of an animal in Group D (40 × 10). Arrow indicates a lesion in which infiltration of inflammatory cells is obvious.

**Figure 5:** A photograph of a longitudinal cochlea slice from an animal in Group C (40 × 10). Arrow indicates a lesion in which “floating cells” are present in the cochlear duct.

**Figure 6:** A photograph of a longitudinal cochlea slice of an animal in Group C (40 × 10). Arrow indicates a lesion in which only some floccules are present in the tympani and no obvious abnormalities can be observed within the inner ear structures.

**Figure 7:** Photograph of a spiral ligament slice of an animal in Group C (40 × 10). Fluorescence reactions were clearly observed, especially in the stria vascularis.

**Figure 8:** Photograph of a longitudinal cochlea slice of an animal in Group C (20 × 10). Significant fluorescence displays were observed in the cochlear bone wall and the lip of the spiral plate.

**Figure 9:** Photograph of a spiral ganglion slice from an animal in Group B (40 × 20). Obvious fluorescence reactions can be observed in ganglion cells.

**Figure 10:** Photograph of a longitudinal cochlea slice from an animal in Group C (10 × 10). Weak coloration was observed in the perivascular modiolus and spiral ganglion.

**Figure 11:** Photograph of a spiral ganglion slice from an animal in Group A (10 × 10). Color reactions were clearly observed in the inner lip of the cochlear bone wall and bone spiral lamina.

**Figure 12:** Photograph of a longitudinal cochlea slice from an animal in Group B (20 × 10). Color reactions were clearly observed in spiral ganglion cells.

**Figure 13:** Photograph of aspiral ganglion slice from an animal in Group A (10 × 10). Color reactions were clearly observed in the perivascular modiolus.

**Figure 14:** Photograph of a semicircular canal transverse slice from an animal in Group A (20 × 10). Color reactions were clearly observed in the ampullary crest.

**Figure 15:** Mitochondrial swelling (arrows) occurred within the epithelial cells of the stria vascularis of an animal in Group C (×30000).

**Figure 16:** Epithelial cells of the stria vascularis with normal morphology in an animal in Group A (×30000).

**Table 1:** Preimmunization, postimmunization, and post-inner-ear-injection antigen-specific antibody levels in serum within each group (*A* value, $\overset{-}{\chi }$  ± *S*).

Group	Preimmunization	Postimmunization	Post-inner-ear-injection
A	0.529 ± 0.125	0.825 ± 0.122	0.814 ± 0.133
B	0.513 ± 0.110	0.818 ± 0.120	0.802 ± 0.141
C	0.531 ± 0.128	0.805 ± 0.118	0.798 ± 0.104
D	0.509 ± 0.122	0.799 ± 0.115	0.779 ± 0.118

Notes

(1) Compared with preimmunization levels, antibody levels in each group (A, B, C, and D) were significantly increased after immunization or after inner ear injection (*t*-test, *P* < 0.05).

(2) Between groups, antibody levels were not significantly different (*t*-test, *P* > 0.05).

**Table 2:** Preimmunization, postimmunization, and post-inner-ear-injection ABR thresholds within each group (dB, sound pressure level) ($\overset{-}{\chi }$  ± *S*).

Group	Preimmunization		Postimmunization		Post-inner-ear-injection	
	Left	Right	Left	Right	Left	Right
A	34.00 ± 5.60	35.00 ± 6.40	69.00 ± 6.60	70.00 ± 6.84	56.00 ± 6.60	49.00 ± 6.70
B	32.00 ± 7.00	33.00 ± 7.20	70.00 ± 8.00	72.00 ± 8.84	60.00 ± 8.00	53.00 ± 7.50
C	36.00 ± 6.30	37.00 ± 5.80	69.00 ± 7.20	68.00 ± 7.52	69.00 ± 7.20	78.00 ± 7.00
D	35.00 ± 7.00	36.00 ± 6.80	68.00 ± 8.50	70.00 ± 9.26	68.00 ± 8.50	69.00 ± 8.00

Notes

(1) Compared with preimmunization ABR thresholds, postimmunization or post-inner-ear-injection thresholds in each group (A, B, C, and D) were significantly increased (*t*-test, *P* < 0.05).

(2) Between groups, ABR thresholds in the left and right ears were not significantly different (*t*-test, *P* > 0.05).
